The article "Effects of Warm Acupuncture Combined with Meloxicam and Comprehensive Nursing on Pain Improvement and Joint Function in Patients with Knee Osteoarthritis" was published in 2022. Journal: J Healthc Eng.

# Effects of Warm Acupuncture Combined with Meloxicam and Comprehensive Nursing on Pain Improvement and Joint Function in Patients with Knee Osteoarthritis

**DOI:** 10.1155/2022/9167956

**Published:** 2022-03-31

**Authors:** Zhengwen Sun, Xiaoli Qu, Tianmei Wang, Feng Liu, Xue Li

**Affiliations:** ^1^Department of Traumatology (I), Yantaishan Hospital, Yantai 264000, China; ^2^Department of Emergency Medicine, Qingdao Eighth People's Hospital, Qingdao 266000, China; ^3^Department of Traditional Chinese Medicine, The Affiliated Qingdao Central Hospital of Qingdao University, The Second Affiliated Hospital of Medical College of Qingdao University, Qingdao 266042, China; ^4^Department of Spine Surgery, Zhangqiu District People's Hospital, Jinan 250200, China; ^5^Department of Spine and Joint, Zhangqiu District People's Hospital, Jinan 250200, China

## Abstract

**Objective:**

To observe the effect of warm acupuncture combined with meloxicam and comprehensive nursing on pain improvement and joint function in patients with knee osteoarthritis.

**Method:**

Eighty-one patients with KOA were randomly divided into control group (CG), traditional Chinese medicine group (TCMG), and combined group (JG). The CG was treated with meloxicam. The TCMG received warm acupuncture treatment. The JG was treated with meloxicam combined with warm acupuncture. Three groups were given comprehensive nursing intervention, and the course of treatment was 4 weeks. Knee function was assessed by knee pain, activity, stability, walking ability, and ability to walk up and down stairs. Improvement time of clinical symptoms of patients was assessed from knee pain, swelling, and movement limitation. Pain mediators (prostaglandin E2 (PGE2), substance P (SP), dopamine (DA), 5-hydroxytryptamine (5-HT)) were detected by enzyme-linked immunosorbent assay (ELISA). Oxidative stress indicators (superoxide dismutase (SOD) and malondialdehyde (MDA)) of the enrolled patients were detected by water-soluble tetrazolium-1 (WST-1) and the thiobarbituric acid (TBA) method. The clinical efficacy was assessed by the visual analog scale (VAS) score.

**Results:**

After treatment, the pain scores of the three groups decreased, and the scores of mobility, stability, walking ability, and the ability to walk up and down stairs increased. Compared with the CG and the TCMG, the JG had a greater range of changes in pain, mobility, stability, walking ability, and ability to walk up and down stairs after treatment. After 7 d, 14 d, and 28 d treatment, PGE2, SP, DA, 5-HT, and MDA in the three groups were decreased compared with before treatment, and the decrease in the JG was more obvious than that in the CG and the TCMG. SOD levels in the three groups were increased, and the increase in the JG was more obvious than that in the CG and the TCMG. The total effective rate of the JG (96.30%) was significantly different from that of the CG (77.78%) and the TCMG (81.48%). The improvement time of knee pain, swelling, and movement limitation in the JG was shorter than that in the CG and the TCMG, and the difference in the improvement time of movement limitation in the TCMG was statistically significant.

**Conclusion:**

Warm acupuncture combined with meloxicam and comprehensive nursing can effectively improve knee swelling and pain in patients with KOA, and the mechanism may be related to reducing the content of inflammatory mediators.

## 1. Introduction

Knee osteoarthritis (KOA) is a common chronic degenerative bone and joint disease in clinic [1]. Its clinical symptoms are mainly knee swelling, difficulty in ascending and descending stairs, knee pain when sitting up, etc. A small number of patients will also show fluid accumulation, pop, etc., which will cause adverse effects on patients' work and life [1]. The incidence of KOA is 8.1% in the middle-aged and elderly population in China, and the incidence of KOA is higher in women than in men, especially after menopause [2]. KOA has become a major cause of disability and reduced quality of life in the elderly. In clinical practice, anti-inflammatory and analgesic conservative treatment is mainly given, but the long-term effect is not obvious, and there are many adverse reactions, resulting in poor tolerance of patients [3, 4]. Therefore, it is very important to find effective treatment measures.

Meloxicam is the main treatment of osteoarthritis that can improve the early symptoms of patients [5]. However, meloxicam has a high incidence of adverse reactions and a high recurrence rate after cure through actual medication [6, 7]. In traditional Chinese medicine (TCM), KOA is classified as “bone paralysis,” and it is believed that the treatment of diseases should focus on the principle of qi and blood, and the principle of equal emphasis on muscles and bones, so as to relieve pain, effectively improve the knee motion and improve the quality of life of patients [8]. Combined with TCM treatment, the patient's body is recuperated while relieving symptoms, so as to improve the overall prognosis. Warm acupuncture has the effect of regulating qi and blood, channelling meridians and activating collaterals, effectively removing wind dampness and stopping arthralgia, and has higher practicability in treating KOA [9, 10]. Clinical practice has found that the implementation of scientific nursing intervention in the treatment of KOA patients can effectively improve the knee function, which is of great significance to promote the recovery of patients and contributes to improve the quality of life of patients [11]. In this study, warm acupuncture combined with meloxicam and comprehensive nursing were used in the treatment of KOA, aiming to provide a reliable basis for the treatment of KOA by integrated Chinese and Western medicine.

## 2. Data and Methods

### 2.1. The General Information

Clinical data of 81 patients with KOA treated in our hospital from January 2020 to January 2021 were retrospectively analyzed, including 47 males and 34 females. The age ranged from 50 to 74 years with an average age of 61.31 ± 6.74 years. The course of disease was 1–5 years, with an average of 2.73 ± 1.37 years. Patients were randomly divided into three groups: control group (CG) with 27 cases, Chinese medicine group (TCMG) with 27 cases, and combined group (JG) with 27 cases. All patients met the diagnostic criteria for KOA. There was no significant difference in general clinical data between the three groups (*P* > 0.05) (Table 1).

### 2.2. Inclusion Criteria and Exclusion Criteria

  Inclusion criteria are as follows: (1) comply with the relevant standards of knee osteoarthritis in guidelines for the diagnosis and treatment of osteoarthritis [12]; (2) patients were diagnosed as knee osteoarthritis by physical examination and imaging examination; (3) signed informed consent; (4) 1 month before receiving treatment, no medication was taken; (5) patient was conscious and able to cooperate with the treatment.
  Exclusion criteria are as follows: (1) allergic; (2) asthma; (3) with mental illness; (4) patients with severe heart failure; (5) digestive ulcer; (6) combined with bone tumor and bone tuberculosis.

### 2.3. Treatment

Patients in 3 groups were treated with symptomatic treatment before medication, such as prohibiting outdoor exercise, ensuring adequate rest, regular diet, good life management, correcting bad habits, and keeping warm.

The CG was treated with meloxicam (national drug approval word H20020217, Shanghai Boehringer Ingelheim Pharmaceutical Co., LTD.), once a day, with warm water after meals, 0.75 mg once. Patients with strong pain can be increased to 1.5 mg.

The TCM group carried out warm acupuncture treatment [13]: choose 1.5 or 2.0 inches filiform needles. For the patients, zusanli, sishencong, neixiyan, waixiyan, yinlingquan, sanyinjiao, dubi, dazhui, weiyang, baihui, fengchi, xuehai, and yintang acupoints are applied with the reinforcing-reducing needling method. After obtaining qi, the moxa column was put on the needle handle, and the column was lit for warm acupuncture treatment once a day in retaining needle within 30 min. After 6 days of treatment, rest for 1 day and 7 days per course of treatment and continuous treatment for 4 courses.

### 2.4. Nursing Methods

Patients in 3 groups were given comprehensive nursing during treatment [14]. (1) Health education: on the basis of understanding the basic information of patients, the etiology, treatment, and precautions of KOA were made into small videos and health knowledge manuals and distributed to patients in the form of ward television, blackboard newspaper column or poster, and detailed disease-related knowledge was explained to them and questions were answered. (2) Psychological guidance: according to the patient's education level and age, the right way to talk with the patient was chosen to understand the patient's inner thoughts. First of all, their ideas are respected and then the patient's psychological problems are put forward. The causes of psychological problems were analyzed to guide the patient to give vent to negative emotions. Patients with good prognosis are invited to exchange their experience. Patients are encouraged to develop hobbies, such as listening to music and reading, to distract attention, and to reduce negative emotions. (3) Dietary guidance: the importance of reasonable diet was emphasized to patients. Coarse grains and fine grains to mix and match were chosen. Patients should eat more fresh fruits and vegetables, quit smoking and alcohol, and avoid spicy and greasy food. (4) Functional exercise guidance: patients were guided to perform passive flexion and extension exercise from passive joint training. The affected limb was fixed on the joint continuous passive motion (CPM) instrument for passive flexion and extension exercise. The initial angle of CPM machine was limited to patient tolerance and then the CPM machine increased by 10° every day and stopped when it reaches a certain angle. Each extension of the knee joint was maintained for 45 s, 30 min/time, 2 times/d, and gradually transitioned to active joint training. Patients was guided to perform muscle training around the knee joint, including the quadriceps exercises (sitting on the bed, taut straight knee joint, slowly lift the affected limb, keep 5∼10 s, repeated practice, 5∼10 min/times, 2∼3 times/d) and hamstring exercise (sitting on the bed, straight the knee joint, knee pressing down on them, for 5 s, repeated practice, 5–10 min/time, 2–3 times/d).

## 3. Observational Index

### 3.1. Improvement Time of Knee Function and Clinical Symptoms

The three groups were compared for knee pain, activity, stability, walking ability, ability to walk up and down stairs, and improvement time of knee pain, swelling, limited activity, and other symptoms.

### 3.2. Clinical Curative Effect

The clinical efficacy was evaluated by the VAS score [15]. (1) Significant effect, VAS score decreased ≥70%; (2) effective, VAS score decreased <70% but ≥30% or higher; (3) invalid, VAS score had no change or decrease <30%. Total efficiency = significant efficiency + effective rate.

### 3.3. Serum Oxidative Stress Index

Superoxide dismutase (SOD) was detected by water-soluble tetrazolium-1 (WST-1), and malondialdehyde (MDA) was detected by the thiobarbituric acid (TBA) method. The kits were purchased from Emjet Technology Co., LTD.

### 3.4. Serum PGE2, SP, DA, and 5-HT Were Detected

In each group, 2 mL venous blood was extracted on an empty stomach in the morning before and after treatment and centrifuged at 4 000 r/min for 10 min. Supernatant was extracted and stored at −80°C for one-time detection after sample collection. The contents of prostaglandin E2 (PGE2), substance P (SP), dopamine (DA), and 5-hydroxytryptamine (5-HT) in serum were detected by enzyme-linked immunosorbent assay (ELISA) in strict accordance with instructions.

### 3.5. Statistical Analysis

SPSS22.0 statistical analysis software was used to analyze the obtained data. All measurement data were represented by $\bar{x}+s$. The *T* test was used to test differences between groups, and count data were measured by the *χ*^2^ test. *P* < 0.05 means the difference is statistically significant.

## 4. Results

### 4.1. Comparison of Knee Function Scores between the Three Groups before and after Treatment

Before treatment, there were no statistically significant differences in pain, mobility, stability, walking ability, and ability to walk up and down stairs among the three groups (Table 2). After treatment, the pain scores of the three groups decreased, while the scores of mobility, stability, walking ability, and the ability to walk up and down stairs increased (Table 2). Compared with the CG and the TCMG, the JG markedly improved in pain, mobility, stability, walking ability, and ability to walk up and down stairs after treatment (Table 2).

### 4.2. Comparison of Pain Mediators among the Three Groups at 0d, 7d, 14d, and 28d of Treatment

There was no significant difference in pain mediators among the three groups on 0 day of treatment (Figure 1). After 7 d, 14 d, and 28 d treatment, PGE2, SP, DA, and 5-HT in the three groups were decreased compared with those before treatment (Figure 1), and the decrease of JG was more obvious than that of CG and TCMG (Figure 1).

### 4.3. Comparison of Clinical Efficacy among the Three Groups

The total effective rate of CG was 77.78% (Table 3). The total effective rate of TCMG was 81.48% (Table 3). The total effective rate of JG was 96.30% (Table 3). For JG, the difference was statistically significant compared with the CG and the TCMG (Table 3).

### 4.4. Comparison of Clinical Symptom Improvement Time among the Three Groups

The improvement time of knee pain, swelling, and activity limitation in the JG was shorter than that in the CG and the TCMG (Table 4); the improvement time of activity restriction in the TCMG was statistically significant compared with the CG (Table 4).

### 4.5. Comparison of Oxidative Stress Index Levels among the Three Groups after 0d, 7d, 14d, and 28d of Treatment

After treatment, there was no significant difference in SOD and MDA levels among the three groups (Figure 2). After 7 d, 14 d, and 28 d treatment, SOD level in all the three groups increased, and the increase in JG was more obvious than that in CG and TCMG (Figure 2). MDA levels in all three groups decreased, and the decrease in JG was more obvious than that in CG and TCMG (Figure 2).

## 5. Discussion

Knee osteoarthritis (KOA) is a common clinical degenerative disease of bone and joint, which can lead to joint deformity or even disability if not treated in time [16]. Meloxicam is a derivative of enolic acid. After acting on the patient's body, meloxicam can quickly enter the blood and directly inhibit the synthesis of inflammatory mediators, including prostaglandins [17, 18]. At the same time, the inhibition intensity of prostaglandin by meloxicam exceeded the biosynthesis ability of kidney and gastric mucosa, which means that patients' healthy tissues will not be affected by the drug and the drug is safe.

In TCM, KOA belongs to the category of “knee paralysis” and “bone paralysis” [8]. The onset of KOA is caused by collateral siltation and stagnant and deficiency of liver and kidney [8]. The treatment is mainly given to promote blood circulation and remove blood stasis, improve dampness, and dissipate cold [8]. Warm acupuncture has obvious curative effect on pain diseases caused by invasion of wind and cold evil qi [9]. Some research results have confirmed that the application of warm acupuncture treatment can improve the clinical treatment effect, relieve the pain of patients, and improve the knee ligament injury [19]. In this study, zusanli, yanglingquan, xiyan, and dubi acupoints were selected for warm acupuncture, among which zusanli was used to treat impotence and paralysis and could supplement the symptoms of deficiency and fatigue; yanglingquan for tendon will point especially lower-limb tendon disease and can shu jin zhuang gu; xiyan is the external meridian acupoint, which has significant effect in the treatment of knee joint pain, joint redness and swelling, leg pain, and weakness; dubi belongs to the liver meridian of foot jueyin, which is the main treatment for knee patella, swelling and pain, cold and wet injection [10].

The comprehensive nursing in this study is comprehensive and covers a wide range, including health education, psychological guidance, dietary guidance, and functional exercise guidance. Health education in comprehensive nursing can explain disease-related knowledge to patients and strengthen their disease cognition so that they actively cooperate with treatment and nursing work. Psychological guidance can alleviate patients' negative emotions and make them establish confidence in treatment. Dietary guidance can promote patients to develop good eating habits and avoid improper diet that affects the effect of disease control. Functional exercise guidance can promote patients to carry out scientific rehabilitation training, which is beneficial to recover their knee function as soon as possible.

Oxidative stress plays an important role in the occurrence and development of KOA. Under normal circumstances, the generating and eliminate of oxygen-free radicals in the body are in a state of balance, and free radicals produced by oxygen metabolism can be cleared in time, and in patients with KOA, oxygen--free radicals generated will increase, excess oxygen-free radical has inhibitory effect on cartilage cell proliferation, can result in cartilage cell aging, and death and thus accelerating the degradation of cartilage matrix, eventually resulting in damage of cartilage [20, 21]. MDA is a product of lipid oxidation and reflects the level of free radicals produced by lipid peroxidation [22]. SOD, as an oxygen-free radical eliminator, can prevent cell lysis and apoptosis, and its level can effectively reflect the antioxidant capacity of the body [23]. The results of this study showed that warm acupuncture combined with meloxicam and comprehensive nursing treatment of KOA can effectively reduce the body's oxidative stress response. In addition, the total effective rate and the improvement time of symptoms such as knee pain, swelling, and movement limitation were also improved after combined treatment. It also shows that warm acupuncture combined with meloxicam and comprehensive nursing is effective in the treatment of KOA. SP is a nociceptive neuropeptide mainly responsible for the transmission of pain information in the body [24]. DA, 5-HT is a peripheral pain medium, which can stimulate sensory peripheral nerves to make the body feel pain [25]. PGE2 can be produced in large quantities in the early stage of inflammation, reduces the pain threshold in the local area of inflammation, and activates the EP receptors on the peripheral sensory nerve endings to enhance the pain sensation [26]. This study found that warm acupuncture combined with meloxicam and comprehensive nursing could significantly reduce the content of pain mediator (PGE2, SP, DA, and 5-HT) in patients with KOA, indicating that meloxicam combined with warm acupuncture has a good analgesic effect.

## 6. Conclusions

Warm acupuncture combined with meloxicam and comprehensive nursing has a clear effect on the treatment of KOA, could improve the clinical symptoms of patients, play a good analgesic effect, and promote patients to recover as soon as possible.

## Figures and Tables

**Figure 1:** Comparison of pain mediators (PGE2 (a), SP (b), DA (c), and 5-HT (d)) in the three groups on 0 d, 7 d, 14 d, and 28 d.

**Figure 2:** Comparison of oxidative stress index levels in the three groups after 0 d, 7 d, 14 d, and 28 d.

**Table 1:** Comparison of general clinical data among the three groups (*n*).

Index	TCMG	CG	JG	*χ* ^2^	*P*
	*n* = 27	*n* = 27	*n* = 27		
Gender					
Female	16	17	14	0.710	>0.05
Male	11	10	13		
Age (years)					
>60	15	16	18	0.723	>0.05
≤60	12	11	9		
Course of disease (years)					
>3	10	9	8	0.333	>0.05
≤3	17	18	19		
Education					
Primary and below	4	5	5	0.602	>0.05
Junior and senior secondary	16	14	16		
Junior college or above	7	8	6		
Pathogenic site					
Left knee	10	12	10	1.818	>0.05
Right knee	9	11	10		
Both knees	8	4	7		

**Table 2:** Comparison of knee function scores between the three groups before and after treatment.

Group	Treatment time	Pain	Mobility	Stability	Walking ability	Ability to walk up and down stairs
CG	BT	78.33 ± 6.41	50.74 ± 5.61	50.93 ± 3.53	59.52 ± 6.12	50.30 ± 3.01
	AT	68.96 ± 6.38	63.30 ± 5.37	58.67 ± 5.34	67.22 ± 7.52	62.93 ± 6.37

TCMG	BT	78.30 ± 6.16	51.37 ± 5.79	50.85 ± 3.47	57.74 ± 6.58	51.37 ± 3.35
	AT	65.89 ± 6.30	66.81 ± 5.94	61.67 ± 5.34	71.37 ± 6.84	65.70 ± 6.37

JG	BT	77.33 ± 6.57	50.44 ± 5.47	51.00 ± 3.57	61.26 ± 6.42	51.30 ± 3.61
	AT	55.89 ± 6.44	74.89 ± 5.51	70.59 ± 7.88	79.19 ± 7.47	69.93 ± 7.20

t0		1.781	2.284	2.066	2.121	1.602
P0		>0.05	>0.05	>0.05	>0.05	>0.05
t1		7.496	7.831	6.512	5.865	3.783
P1		<0.05	<0.05	<0.05	<0.05	<0.05
t2		5.769	5.181	4.874	4.008	2.283
P2		<0.05	<0.05	<0.05	<0.05	<0.05

*Note.* BT: before treatment; AT: after treatment; T0, P0: the comparison between the CG and the TCMG after treatment; T1, P1: the comparison between the CG and the JG after treatment. T2, P2: the comparison between the TCMG and the JG after treatment.

**Table 3:** Comparison of clinical efficacy among the three groups.

Group	*n*	Significant effect	Effective	Invalid	Total effective rate
CG	27	11	10	6	21 (77.78)
TCMG	27	13	9	5	22 (81.48)
JG	27	22	4	1	26 (96.30)
*χ* ^2^0					0.310
P0					>0.05
*χ* ^2^1					9.810
P1					<0.05
*χ* ^2^2					6.904
P2					<0.05

*Note. χ* ^2^0, P0: the comparison between the CG and the TCMG; *χ*^2^1, P1: the comparison between the CG and the JG; *χ*^2^2, P2: the comparison between the TCMG and the JG.

**Table 4:** Comparison of improvement time of clinical symptoms among the three groups.

Group	*n*	Improvement time of clinical symptoms/d		
		Knee pain	Swelling	Activity limitation
CG	27	15.44 ± 1.12	8.96 ± 0.81	19.59 ± 1.12
TCMG	27	14.96 ± 0.85	8.48 ± 1.05	18.44 ± 1.12
JG	27	8.93 ± 0.78	5.93 ± 0.83	10.89 ± 0.85
t0		1.775	1.887	3.768
P0		>0.05	>0.05	<0.05
t1		24.790	13.640	32.230
P1		<0.05	<0.05	<0.05
t2		27.110	9.920	27.940
P2		<0.05	<0.05	<0.05

*Note.* T0, P0: the comparison between the CG and the TCMG; T1, P1: the comparison between the CG and the JG; T2, P2, the comparison between the TCMG and the JG.

## Data Availability

Data used to support the findings of this study are available on reasonable request from the corresponding author.
